# Construction of Community Medical Communication Service and Rehabilitation Model for Elderly Patients under the Internet of Things

**DOI:** 10.1155/2022/9689769

**Published:** 2022-03-29

**Authors:** Xiaoxia Zhang, Fang Wang, Dan Wang, Yanhua Xiang, Zhongwei Zhang

**Affiliations:** ^1^Changsha Social Work College, Changsha, Hunan, China; ^2^Dongfang Electric Corporation, Chengdu, Sichuan, China

## Abstract

The objective of this study was to discuss the health management of elderly patients in the community and the management of community rehabilitation under the support of the new Internet of Things (IoT). The IoT technology was adopted to monitor the wearable devices through mobile medical physiological data. The heart rate, blood pressure, respiratory rate, and other physiological indicators of the elderly were collected in real time. The support vector machine (SVM) algorithm was selected as the core algorithm for the elderly physiological index disease risk assessment, the fuzzy comprehensive evaluation method was adopted as the core method of the elderly disease risk quantitative assessment model to process the physiological indicators, and finally, a reasonable physiological index processing model and quantitative indicators of disease risk were obtained. The data on vascular disease were selected from the MIMIC database. In addition, the advantages and disadvantages of the SVM algorithm and the Backpropagation Neural Network (BPNN) algorithm were compared and analysed. The final verification results showed that the fusion accuracy of the SVM processing MIMIC database and the University of California Irvine (UCI) dataset was 0.8327 and 0.8045, respectively, while the fusion accuracy of the BPNN algorithm in processing the same data was 0.7792 and 0.7288, respectively. It was obvious that the fusion accuracy of the SVM algorithm was higher than that of the BPNN algorithm, and the accuracy difference of the SVM algorithm was lower than that of the BPNN algorithm in different groups of data. In the verification of the elderly disease risk quantitative assessment model, the results were consistent with the selected data, which verified the effectiveness of the design model in this study. Therefore, it can be used as a quantitative assessment model of general elderly physiological indicators of disease risk and can be applied to the community medical communication management system. It proved that the model of medical communication and rehabilitation services for elderly patients in the community constructed in this study can definitely help the development of community service for the elderly.

## 1. Introduction

With the development of society, the aging society has become an important social problem that most countries inevitably need to face [1]. According to relevant investigations and studies, as of the end of 2019, the number of elderly people aged 60 and over in China totalled 253.88 million as of the end of 2019, accounting for 18.1% of the total population of the country, of which, there are 176.03 million people aged 65 and over, accounting for 12.6% of the total population of the whole country. Compared with 17.9% of the elderly population aged 60 and above in 2018 and 17.3% in 2017, the current aging trend is becoming increasingly severe [2–4]. With the gradual severity of the aging problem, there are currently 37,021 legally registered and licensed elderly care institutions in China as of the end of 2019, with a total of 4.674 million beds. It means that the vast majority of elderly people find it difficult to enjoy the services of social public elderly care, and they are more dependent on families and individuals. According to the latest survey, the family pension model for the elderly in 2020 is still not the current main pension model, accounting for 90% of the national pension, while the institutional pension and the community pension account for only 7% and 3%, respectively. This data are especially highlighted in the vast rural areas [5]. The incidence of chronic diseases and malignant tumours increases with age. After illness, the probability of complications increases significantly, making the disease management and prognosis of the elderly extremely complicated and slow in progress [6–8]. Therefore, it is difficult to meet the actual needs of the elderly simply by family support, and community support has become the best solution at present. It not only satisfies the “acquaintance” environment pursued by the elderly but also allows the community to provide relatively professional management of the elderly, and it can give full play to the advantages of grassroots management in China [9–12].

Community elderly care mainly introduces elderly care services into the community so that the elderly can provide for the elderly at home. It not only respects the willingness of the elderly to provide for elderly care at home but also combines the professionalism and convenience of social elderly care. It is a new and characteristic elderly care method for the aging society in China. Community care and elderly care services are gradually established through government supervision, social participation, and market management. The community service for the elderly, with family care as the core, community services as the support, and professionalism as the guide, is to provide the elderly care services in all aspects of daily life, health management, spiritual civilization, and cultural entertainment. The development of various convenient services is inseparable from the role of communication terminal equipment for the elderly and the intelligent platform for the elderly in the community [13–16].

Internet of Things (IoT) refers to the collection of information through various sensors, real-time collection of any required information, and transmission through the Internet to achieve a wide range of connections among objects and people and objects and to achieve intelligent identification and connection of objects [17]. In layman's terms, IoT is based on the Internet through smart devices to realize the collection and artificial intelligence processing of surrounding objects and various types of information. In China, IoT has long been widely used in smart cities, traffic diversion, environmental remediation, government work, social stability, logistics and transportation, smart homes, industrial production, campus life, food safety, public services, life and health, and personal care [18]. The development of IoT is not only a demand of society but also a demand for people who aspire to make life more convenient in the future [19–21].

With the continuous deepening of IoT technology in the health field, the continuous reform and innovation of wearable devices function so that they can fully meet the current technical needs of the health and rehabilitation management of the elderly. Applying this technology to the health management of elderly patients in the community can solve the inconvenience, psychological resistance, and long-term continuous physiological monitoring of elderly patients and can locate and notify community personnel and medical staff in a timely manner under abnormal physiological conditions. Some elderly people can communicate and supervise the rehabilitation information. It makes up for the lack of community care for the health management of the elderly and improves the monitoring of the physiological conditions of the elderly by the community and medical staff. In the case of not affecting the normal life of the elderly as much as possible, managing the physical health of each elderly person has played a key auxiliary role in community elderly care [22–24].

In summary, the aging of the population is currently a major problem facing the country and society. How to meet the needs of the elderly and society needs to be solved urgently. Therefore, this work discusses the health management of elderly patients in the community and the support of the new Internet of Things. The application of community rehabilitation management is different from previous studies. This work uses the popular Internet of Things technology in recent years, combines community medical services for elderly patients, and adopts intelligent electronic equipment to realize automated monitoring of various physiological indicators of elderly patients, with a view to providing new strategies for the rehabilitation management of elderly patients in the community.

## 2. Technologies and Methods

### 2.1. Wearable Devices

With the advent of Google Glass in 2012, the “first year of smart wearable devices” also kicked off. Nowadays, with the commercial application of high-precision sensors, wearable devices have long been used in the daily lives of most people. The common sports bracelets, smartwatches, smart rings, smart glasses, and smart gloves generally have requirements for biometric identification, such as long-term continuous monitoring of electrocardiogram, body temperature, blood pressure, heart rate, and blood oxygen. At present, the domestic wearable devices market is mainly concentrated in major Internet manufacturers such as Huawei, Xiaomi, Apple, and OV. According to the China Wearable Devices Market Quarterly Tracking Report, the Fourth Quarter of 2020, released by Internet Data Center (IDC) data agency, the wearable devices market shipments in the fourth quarter of 2020 were 30.26 million units in China, with a year-on-year increase of 7.7%. Among them, basic wearable devices were 25.18 million units, with a year-on-year increase of 10.3%, and smart wearable devices were 5.08 million units, with a year-on-year decrease of 3.6%. In foreign markets, Apple still tops the list with 55.6 million units, with a market share of 36.2%, followed by Xiaomi with 13.5 million units, with a market share of 8.8%, and then followed by Samsung with 13 million units and Huawei 10.2 million units. The continuous hot industry growth has never stopped the development of technology.

### 2.2. Construction on Community Medical Communication Service and Rehabilitation Model

With the continuous upgrading of wireless sensing technology in wearable devices in recent years, the accuracy and stability of physiological data monitoring of the human body have gradually increased [25]. For elderly patients, the daily records of physiological indicators such as blood pressure, blood sugar, heart rate, weight, and sleep quality are very important. These data not only reflect the current physical health of the elderly but also can predict future physical health. In traditional elderly care services, it is often necessary for the elderly to go to the community for testing or community personnel to collect data daily, which is time-consuming and laborious and cannot achieve the effect of real-time monitoring. Introducing wearable devices into community pensions and applying IoT technology to the health monitoring of the elderly can solve the above problems. The community elderly medical information supervision system is shown in Figure 1.

### 2.3. IoT Technology

IoT refers to the collection of information through various sensors and real-time collection of any required information and transmission via the Internet to achieve a wide range of connections among objects, people, and objects and to achieve intelligent identification and connection of objects. IoT can be roughly divided into a three-tier architecture, including information collection, data transmission, and smart port. Information collection mainly comes from the real-time collection of peripheral information by various sensors, periodically obtaining the required information and continuously updating and classifying the collected data. Data transmission is the real-time transmission of collected data through various wired or wireless networks to ensure information security and data accuracy during the transmission process. It is the most core technology in the entire IoT technology link. The smart port is a port for IoT to interact with enterprises and individuals. It can transmit the collected data to the user interface and perform personalized processing so that it can meet the needs of users and finally implement the personalized smart applications of the IoT.

Sensor technology refers to a chip or device that can stably sense and convert the monitored information into a signal that can be transmitted according to a certain logic. Nowadays, the requirements for sensors are not satisfied with the general data transmission, and a certain amount of intelligent processing is needed. It needs to have a certain degree of self-adaptation to the changes of external information and be able to perform data preprocessing and diagnosis.

Embedded technology refers to a system or software that is controlled by an internal computer to perform personalized customization functions. The embedded system is completely customized for the specific role of the user. It is mostly composed of a microcontrol module, a nonvolatile read-only memory module, a volatile random access memory module, a sensor module, an analog-to-digital conversion module, a control module, a display module, and a lightweight embedded operating system. Among them, the monolithic microcontroller is the core of most embedded systems.

### 2.4. Electronization of Elderly Ability Assessment

The Elderly Ability Quantitative Table is a subjective quantitative evaluation system for the elderly to assess their own abilities. After the electronization, it not only saves the dependence on paper quality but also facilitates the update and retention of evaluations in the future, facilitates the elderly to fill in anytime and anywhere, and reduces the workload of the elderly and community workers.

For the selection of the scale, the Abilities Assessment of the Elderly issued by the MCA is undertaken as the basis of the scale. The assessment refers to the ability assessment system for the elderly in Europe, America, and surrounding areas of China, Taiwan, and Hong Kong and establishes the ability of the elderly to evaluate the content and corresponding grades with Chinese characteristics.

The Elderly Ability Assessment scale is divided into 4 first-level indicators in this study, and the first-level indicators are graded into 25 second-level indicators. The specific items are shown in Table 1.

Each grade is divided into three levels: 0 points require great assistance from others or complete assistance from others; 5 points require partial assistance from others or rarely require assistance from others; and 10 points can be completed independently. Each level indicator has a corresponding score coefficient, and the basic coefficient is 0.5. For some basic ability indicators such as walking on flat ground, holding and placing, and level of consciousness, the coefficient needs to be increased to 1. The final score and other vector data are filed together with the community medical workstation, and the specific value is judged by the medical staff.

### 2.5. Monitoring Technology of Physiological Indicators

At present, there are relatively mature and commercial high-precision sensors all over the world, which can continuously monitor electrocardiograph (ECG), body temperature, blood pressure, heart rate, blood oxygen, and other parameters for a long time. In addition, the high-precision sensors have been applied to wearable devices for commercialization and integrate the global position system (GPS) positioning and Wireless Fidelity (Wi-Fi) module.

Photoplethysmography (PPG) is commonly used at present. This technology irradiates the skin. Because blood is highly impermeable, it will reflect red light and absorb green light. The reflected light is collected by the sensor through projection or reflection, converted into electrical signals, and converted into PPG through corresponding processing. The principle is shown in Figure 2.

In Figure 2, *X* is the incident light intensity, *X*_max_ is the maximum output light, and *X*_min_ refers to the minimum output light. According to the Lambert-Beer law between blood composition and absorbance, equation (1) can be obtained:

(1) $$\begin{array}{c} \Delta Y^{\lambda }=\mathrm{lg}\frac{X_{O}^{\lambda }}{X_{\min}^{\lambda }\mathrm{lg}\left(X_{O}^{\lambda }/X_{\max}^{\lambda }\right)}. \end{array}$$

In the above equation, Δ*Y*^*λ*^ refers to the absorbance of pulsating arterial blood at the wavelength *λ*; *X*_*O*_^*λ*^, *X*_max_^*λ*^, and *X*_min_^*λ*^ represent the intensity of the incident light, the maximum output light, and the minimum output light, respectively. Equation (1) can be simplified to equation (2).

(2) $$\begin{array}{c} \Delta Y^{\lambda }=\sum_{x}^{n}\varepsilon_{x}\cdot c_{x}\cdot l. \end{array}$$

In equation (2), *ε*_*x*_, *c*_*x*_, and *l* represent the molar extinction coefficient and concentration of the *x*-th component in the blood and the equivalent optical path length of the pulsating blood in the maximum filling state, respectively.

The wearable device collects human body-related data through sensors and performs PPG processing, which can directly obtain physiological data such as heart rate, blood pressure, and pulse that are required for daily monitoring.

### 2.6. GPS Positioning

In this experiment, the geographic location of the elderly wearing is displayed on the map in real time by connecting to the open API interface of AutoNavi Map. The three-axis acceleration sensor is adopted to collect the changes in the wearer's spatial position and sudden spatial changes such as falling and violent exercises. In addition, specific elderly people are dealt with accordingly.

The specific working principle of the three-axis acceleration sensor is shown in Figure 3. It can be judged whether the wearer is in a spatial abnormal state by monitoring the position values in the *X*, *Y*, and *Z* directions of the coordinate axis.

### 2.7. Radio Technology

Wearable monitoring devices can currently use Bluetooth, ZigBee, Wi-Fi, and mobile communication mainstream transmission methods. Among them, Bluetooth is suitable for short-distance high-speed transmission, but its power consumption and cost are relatively high. ZigBee is suitable for short-distance, low-latency, low-power, and high-security transmission protocols. It is currently mainly used in various short-distance mechanical control, medical, home intelligent control, and other fields. Wi-Fi is suitable for the construction and wireless connection of mobile networking in a small area. The mobile communications (3G, 4G, 5G, etc.) are suitable for large-scale high-speed and high-quality communications.

### 2.8. Analysis of Physiological Indicators for Elderly Patients

Based on the initial analysis of the physiological indicators of the elderly in the community, the community health information files are established and classified, and all the physiological indicators of the elderly can be studied. The specific mode is shown in Figure 4.

The data of physiological indicators for the elderly in the community can be undertaken as a benchmark to learn and train the support vector machine (SVM). SVM is a common method to solve data classification and analysis. It uses the optimal hyperplane in data classification and processes two-dimensional linear inseparable samples through the high-dimensional mapping of the kernel function to obtain the global optimal solution.

The fuzzy comprehensive evaluation method (FCEM) is used as the evaluation method for the physiological indicators of the elderly group for abnormal tendency. Determining the index weight and selecting the membership function are the most critical technical issues.

For the index weight, principal component analysis (PCA) is selected as the method of determination. PCA combines *x* physiological indicators with certain connections to form *n* independent parameters to replace the original indicators. Its mathematical model is shown in equation (3).

(3) $$\begin{array}{c} \left\{\begin{array}{c} M_{1}=a_{11}Z_{1}+a_{21}Z_{2}+\cdots +a_{x1}Z_{x},\\ M_{2}=a_{12}Z_{1}+a_{22}Z_{2}+\cdots +a_{x2}Z_{x},\\ \ldots \\ M_{n}=a_{1n}Z_{1}+a_{2n}Z_{2}+\cdots +a_{xn}Z_{x}. \end{array}\right. \end{array}$$

In equation (3), *M* is the principal component, with a total of *n* groups, where *a*_11_ … *a*_*xn*_ represent the eigenvector corresponding to the eigenvalue of the original data Z(*Z*_1_, *Z*_2_,…, *Z*_*x*_) covariance matrix and *Z*_1_ … *Z*_*x*_ represent the normalized vector of the data. The principal component contribution rate can be calculated with the following equation:

(4) $$\begin{array}{c} f_{n}=\frac{\sum_{q-1}^{n}\lambda_{q}}{\sum_{q-1}^{x}\lambda_{q}}\;\left(n=1,\ldots ,x\right). \end{array}$$

It is assumed that the contribution rate *f*_1_ + *f*_2_ corresponding to the first and second principal components *M*1 and *M*2 > 85% and the pair of *M*1 and *M*2 can describe the original information. Regarding its weight, it can be calculated with the following equation:

(5) $$\begin{array}{c} g_{1}=\frac{a_{11}f_{1}+a_{12}f_{2}}{f_{1}+f_{2}}. \end{array}$$

Similarly, the *g*_*n*_ weight equation is shown as follows:

(6) $$\begin{array}{c} g_{n}=\frac{a_{n1}f_{1}+a_{n2}f_{2}}{f_{1}+f_{2}}. \end{array}$$

In this study, the *K*th parabolic function is selected as the membership function of the risk level, which can be calculated with the following equations:

(7) $$\begin{array}{c} T\left(x\right)=\left\{\begin{array}{cc} 1, & x<a,\\ {\left(\frac{b-x}{b-a}\right)}^{k}, & a\leq x\leq b,\\ 1, & b\leq x, \end{array}\right. \end{array}$$

(8) $$\begin{array}{c} T\left(x\right)=\left\{\begin{array}{cc} 0, & x<a,\\ {\left(\frac{x-a}{b-a}\right)}^{k}, & a\leq x\leq b,\\ 1, & b<x, \end{array}\right. \end{array}$$

(9) $$\begin{array}{c} T\left(x\right)=\left\{\begin{array}{cc} {\left(\frac{x-a}{b-a}\right)}^{k}, & a\leq x\leq b,\\ {\left(\frac{d-x}{d-c}\right)}^{k}, & c\leq x\leq d\\ 0, & x<a,d<x. \end{array}\right. \end{array}$$

Equation (7) is small-sized, equation (8) is medium-sized, and equation (9) is large-sized; *a*, *b*, *c*, and *d* are the four types of indicators for the analysis and evaluation of the specific physiological indicators of elderly patients. The model is shown in Figure 5.

In the process, the collected data has to be preprocessed firstly. The min–max normalization in the linear method is adopted in the normalization process in this study, which is specifically shown in equation (10):

(10) $$\begin{array}{c} x^{*}=\frac{x-a}{b-a}. \end{array}$$

In the equation above, *a* is the minimum value in the sample data, and *b* is the maximum value in the sample data.

Attribute reduction is to eliminate repetitive and useless attributes through algorithms so that the reduced subset can get the same attribute results as the original conditions. The steps are shown in Figure 6.

(11) $$\begin{array}{c} f\left(x\right)=k\left(1-\frac{\text{card}\left(x\right)}{n}\right)+\left(1-k\right)\frac{\gamma_{c^{`}}\left(D\right)}{\gamma_{C}\left(D\right)}. \end{array}$$

In equation (11), card(x) is the number of particle attributes, *n* is the total number of attributes, *γ*_*c*^`^_(*D*) is the particle dependency, *γ*_*c*_(*D*) is the dependency of the total set of attributes under the original conditions, and *k* refers to a self-defined parameter. If more sensitive information is calculated, it should appropriately reduce *k*; and if fewer attributes are required, it can increase the value of *k* appropriately.

### 2.9. Attribute Reduction and Parameter Optimization Based on Improved PSO-SVM

Particle swarm optimization (PSO) is a population-based stochastic optimization technology that optimizes the accuracy of the parameters in the SVM algorithm by selecting the PSO algorithm so as to improve the accuracy of the vector machine for grading and evaluating the abnormal physiological parameters of the elderly. The specific process is shown in Figure 7.

### 2.10. Verification Experiment of Fusion Algorithm

The data of 90 patients from the MIMIC database, Numeric/055n database, and 180 patients with vascular disease from the UCI database were randomly selected as the verification data for algorithm verification. The Backpropagation Neural Networks (BPNN) algorithm is adopted to verify the SVM algorithm used in this study. The database data are fused, and the fusion accuracy is judged to determine the pros and cons of the SVM algorithm and the BPNN algorithm.

### 2.11. Fuzzy Comprehensive Assessment of Disease Risk

Due to the high coupling and nonlinear relationship of physiological indicators, disease risk assessment mainly relies on the subjective judgment of professional knowledge and experience of medical staff. The fuzzy comprehensive assessment is adopted as a quantitative assessment method of disease risk in the elderly, and the fuzzy membership function and fuzzy product rule are selected to simulate the medical staff system and professional knowledge in this study.

The fuzzy relationship matrix is represented by *F* (*F*_1_, *F*_2_,…, *F*_*n*_), and its specific relationship is shown in equation (12):

(12) $$\begin{array}{c} F=\left\{\begin{array}{c} F_{1}\\ F_{2}\\ \ldots \\ F_{n} \end{array}\right\}=\left[\begin{array}{cccc} f_{11} & f_{12} & \ldots & f_{1n}\\ f_{21} & f_{22} & \ldots & f_{2n}\\ \ldots & \ldots & \ldots & \ldots \\ f_{x1} & f_{x2} & \ldots & f_{xn} \end{array}\right]. \end{array}$$

Here, *n* is the number of influencing factors, and *x* refers to the evaluation level. *B* is defined to be the set of evaluation value vectors in the evaluation set, and *B* represents the probability of a certain risk level and the degree of occurrence at this level. The equation is as follows:

(13) $$\begin{array}{c} B=A\circ F=\left(a_{1},a_{2},\cdots ,a_{x}\right)\circ \left[\begin{array}{cccc} f_{11} & f_{12} & \ldots & f_{1n}\\ f_{21} & f_{22} & \ldots & f_{2n}\\ \ldots & \ldots & \ldots & \ldots \\ f_{x1} & f_{x2} & \ldots & f_{xn} \end{array}\right]. \end{array}$$

In equation (13), *A* refers to the weight vector *A* = (*a*_1_, *a*_2_,…, *a*_*x*_) (0 ≤ *a*_*i*_ ≤ 1, *i* = 1,…, *x*), and ∘ is the operator. *M*(*·*, ⊕) is selected for operation in this study. The specific algorithm is shown in equation (14):

(14) $$\begin{array}{c} U_{c}=\min\left(1,\sum_{t-1}^{x}a_{t}f_{tc}\right). \end{array}$$

In equation (14), *U*_*c*_ represents the membership degree of the graded fuzzy subset *r*_t_ in the fuzzy comment set *R* for evaluating disease risk, *c* = 1, 2,…, *n*, *·* is a real number operation, and ⊕ refers to the sum operation up to 1.

The final risk level is to avoid losing too much information and getting wrong information. The weighted average principle is adopted to calculate the number of cases as follows:

(15) $$\begin{array}{c} j^{*}=\frac{\sum_{i=1}^{x}\mu \left(r_{i}\right)\cdot u_{i}}{\sum_{i=1}^{x}u_{i}}. \end{array}$$

In equation (15), *μ*(*r*_*i*_) is the evaluation grade value variable, with the principle of maximum membership *U*=max{*u*_1_, *u*_2_,…, *u*_*i*_}. In the end, the risk value of a certain factor influencing the elderly's illness is calculated as shown in equation (16):

(16) $$\begin{array}{c} f=\frac{0.5}{L-M}\times \left(\text{cur\_val }-M\right)+0.5. \end{array}$$

In the equation above, *L* represents the maximum value of factor risk, corresponding to fuzzy risk level 1; *M* refers to the median value of factor risk, corresponding to fuzzy risk level 0.5; and cur_val represents the current measured value of the factor.

### 2.12. Examples of Quantitative Disease Risk Assessment

A case of data from the MIMIC database, Numeric/055n, is selected as a model for elderly disease risk assessment in the community based on fuzzy comprehensive assessment. The specific data used is shown in Table 2.

This model is brought into the above-mentioned physiological indicators risk assessment model for the elderly. Firstly, its membership function is determined, and then a fuzzy matrix is constructed based on the fuzzy value of each influencing factor. The fuzzy comprehensive score is calculated from the fuzzy relationship and the weight matrix. According to the principle of nearest neighbour value, the risk level of elderly disease is judged.

### 2.13. Family Health Self-Management

Family health self-management is an important connection part between elderly patients and medical staff and between family and community medical workstations. The above-mentioned system is adopted to assess the health risks of elderly patients. Medical staff receive the information on risk factors, conduct real-time and continuous online monitoring of health conditions, and then provide targeted health advice and guidance for elderly patients. For elderly patients with higher health risks, medical staff can take targeted health interventions to help them deal with health matters.

In addition, real-time communication and video chat are also important means to protect the physical and mental health of elderly patients. Based on real-time communication, it can grasp the physical and mental conditions of elderly patients, provide health interventions and guidance (including correction of bad living habits and eating patterns), and provide mental health guidance and spiritual comfort. It can give full play to the advantages of traditional Chinese medicine (TCM) in “preventing disease,” suggest targeted treatments such as medicated diet to elderly patients, provide targeted rehabilitation training and guidance to elderly patients in need of rehabilitation, and give corresponding supervisions.

For elderly patients living alone at home, a one-button call for help function is provided, equipped with the GPS system, to facilitate timely call for help to community medical institutions when needed.

### 2.14. Construction of Community Medical Workstation

Community medical workstations take IoT as the core and play a role as a link among elderly patients, communities, and hospitals. The workstation monitors the physiological indicators of the elderly in the community on a daily basis and establishes long-term electronic information files for the elderly. In addition, the health risk assessment feedback from the intelligent system is verified and further analysed, and targeted health interventions are made for elderly patients to provide professional physical, psychological, and social support. If required by elderly patients, they can consider providing further on-site services or contacting an ambulance.

### 2.15. Training of Medical Personnel

As the community undertakes the health management of elderly patients, the shortage of grassroots medical personnel has become an important factor restricting the development of community care for the elderly. In response to the rapid increase in the incidence of chronic diseases in elderly patients, community medical staff are more inclined to health prevention, health management, and rehabilitation. In order to solve the current shortage of community medical personnel, lack of professionalism, and irrational distribution of personnel, a training mechanism that integrates medical care and maintenance should be adopted. For community medical stations, relevant government departments propose targeted training norms and the transformation of in-service personnel. It can cultivate relevant technical professionals in colleges and technical schools to engage in community health management services for elderly patients and provide follow-up learning and promotion channels.

## 3. Results and Discussion

### 3.1. Comparison Results of Fusion Algorithms

The selected two sets of physiological data are fused on SVM and BPNN, respectively, and the fusion accuracy is shown in Figure 8.

As given in Figure 8, the SVM algorithm is generally higher than the BPNN algorithm from the overall fusion accuracy point of view; the difference of SVM algorithm in different data fusion results is 0.0282, while the difference of BPNN algorithm is 0.0504 in terms of fusion results. This proves that the SVM algorithm is better than the BPNN algorithm in overall fusion accuracy. When different results are processed, the SVM algorithm fusion results show less difference, indicating that the SVM algorithm has reduced dependence on typical samples; in this study, selection data are common due to the study of elderly patients in the community. For special patients, targeted observation is adopted, which is not within the scope of home monitoring. Therefore, the SVM algorithm is more suitable for the construction of the algorithm used in this study.

Tafreshi. et al. [26] used fuzzy algorithms to reduce the false alarm rate of blood pressure and ECG monitors, which can measure the blood pressure-ECG delay. Mainardi et al. [27] proposed a bipartite interpolation recursive identification model for the measurement of beat-to-beat parameters, which helps describe and detect the heart rate, arterial blood pressure, and neuromodulation of the patients. Tashiro et al. [28] proposed the use of neural network algorithms for the independent recognition of high-frequency ECG signals. This method can reduce the transfer of samples between high-frequency ECG and neural network algorithms, effectively optimizing the data recognition accuracy and classification efficiency.

### 3.2. Results of Quantitative Disease Risk Assessment

The risk level is set as *F* = {*f*_1_, *f*_2_, *f*_3_}, which are high-risk, low-risk, and health, respectively. Their level fuzzy value is *F* = {0.9, 0.5, 0.1}. According to the physiological indicators risk quantitative assessment model for the elderly, *f*_1_∼*f*_3_ are introduced in the fuzzy membership function, *k* is set to 1.1, and its function is as follows:

(17) $$\begin{array}{c} T_{1}\left(x\right)=\left\{\begin{array}{cc} 1, & x>0.9,\\ {\left(\frac{x-0.5}{0.4}\right)}^{1.1}, & 0.5\leq x\leq 0.9,\\ 0, & x\leq 0.5, \end{array}\right. \end{array}$$

(18) $$\begin{array}{c} T_{2}\left(x\right)=\left\{\begin{array}{cc} 0, & x<0.1,\\ {\left(\frac{x-0.1}{0.35}\right)}^{1.1}, & 0.1\leq x\leq 0.45,\\ 1, & 0.45\leq x\leq 0.55,\\ {\left(\frac{0.9-x}{0.35}\right)}^{1.1}, & 0.55\leq x\leq 0.9,\\ 0, & x\geq 0.9, \end{array}\right. \end{array}$$

(19) $$\begin{array}{c} T_{3}\left(x\right)=\left\{\begin{array}{cc} 0, & x>0.5,\\ {\left(\frac{0.5-X}{0.35}\right)}^{1.1} & 0.1\leq x\leq 0.5,\\ 1, & x<0.1. \end{array}\right. \end{array}$$

Equations (17)∼(19) are fuzzy membership functions *f*_1_∼*f*_3_. All influencing factors are processed according to the fuzzy calculation model, and the fuzzy value of the risk degree of each factor is obtained, which are 0.59, 0.25, 0.42, 0.76, 0.91, and 0.27, respectively. According to the above results, the membership function is introduced to construct a fuzzy relationship matrix, and then according to the weight vector, the quantitative risk assessment results of the elderly physiological indicators are judged. The fuzzy relation matrix is shown in equation (18):

(20) $$\begin{array}{c} F=\left[\begin{array}{ccc} 0.211 & 0.795 & 0\\ 0 & 0.38 & 0.54\\ 0 & 0.929 & 0.123\\ 0.649 & 0.276 & 0\\ 1 & 0 & 0\\ 0 & 0.44 & 0.486 \end{array}\right]. \end{array}$$

The six parameters of the selected data in the MIMIC database, Numeric/055n database, are used for the PCA, and the weights of these six influencing factors are calculated. Part of the data in the database is shown in Table 3.

The physiological indicators data are normalized, and then their characteristic values and contribution rates are calculated. The results are shown in Table 4.

The first two rows of data are undertaken as the main parameters to build the principal component model:

(21) $$\begin{array}{c} \left\{\begin{array}{c} T_{1}\left(x\right)=0.2634x_{1}+0.2393x_{2}+0.2445x_{3}-0.1334x_{4}+0.085x_{5}+0.2571x_{6},\\ T_{2}\left(x\right)=0.1668x_{1}+0.3816x_{2}-0.2337x_{3}+0.6967x_{4}-0.3876x_{5}+0.1882x_{6}. \end{array}\right. \end{array}$$

In equation (21), *x*_1_∼*x*_6_ are the six related parameters in Table 3 except risk grade. The weight value of each parameter can be calculated according to equation (21) to obtain the weight vector *Q*:

(22) $$\begin{array}{c} Q=\left(0.2421,0.2723,0.1332,0.0611,0.0276,0.2409\right). \end{array}$$

According to the weight vector, the fuzzy evaluation value *A* is calculated according to equation (13):

(23) $$\begin{array}{c} A=Q\circ F=\left(0.119,0.549,0.283\right). \end{array}$$

In the equation above, *F* is the fuzzy relationship matrix of equation (18), and the membership level *j∗* is calculated by the weighted average principle according to equation (15):

(24) $$\begin{array}{c} j^{*}=\frac{\sum_{i=1}^{x}\mu \left(r_{i}\right)\cdot u_{i}}{\sum_{i=1}^{x}u_{i}}=\frac{0.119\times 0.9+0.549\times 0.5+0.283\times 0.1}{0.119+0.549+0.283}=0.431. \end{array}$$

If the calculated membership grade of 0.431 is near 0.5 in the comment concentration, it means that the disease risk factor of the physiological indicators is 0.5 (low risk), which is consistent with the sample grade label 2 (low risk) of the data in the MIMIC database, Numeric/055n database. It shows that the fuzzy comprehensive evaluation model based on the PCA method provided in this study is effective and can be used for the quantitative evaluation of the disease risk of normal elderly physiological indicators.

Tonekabonipour et al. [29] compared and verified the fuzzy neural algorithm and the network neural algorithm in the accuracy of ECG processing, and the results showed that the fuzzy neural algorithm is superior to ECG. Lai et al. [30] believed that the SVM combined with particle swarm optimization (PSO) algorithm has greatly improved the accuracy of classification and recognition and general application compared with other classification methods.

## 4. Conclusion

Based on the IoT, a model of medical communication and rehabilitation service is constructed for elderly patients in the community in this study. On the basis of mobile communication medical testing wearable devices, artificial intelligence is used to monitor elderly physiological indicators, quantitatively evaluate disease risks, and complete long-term and continuous monitoring of the physical condition of the elderly in the jurisdiction by the community. In addition, it helps community medical stations to carry out rehabilitation service and daily health management for elderly patients. Based on the existing basis, the physiological data of the human body are combined with the SVM by analysing physiological parameters, GPS, and other data to design a reasonable physiological indicator processing model and disease risk quantitative indicators. The quantitative relationship between six physiological indicators and disease risk is analysed, and the dimensionality of feature attributes is reduced to improve the quantum swarm algorithm to obtain the best combination of parameters and finally verify the effectiveness of the model through testing. The results suggested that the SVM algorithm showed better fusion accuracy and lower accuracy difference. Therefore, the community-based medical communication and rehabilitation service model for elderly patients constructed in this study was definitely helpful to the development of community services for the elderly. However, when the model is built, a single physiological factor is considered only in this study, and it fails to consider some special diseases such as upper and lower limb disabilities. In the construction of the disease risk quantitative assessment model, the accuracy can still be further classified. It is believed that, with the continuous growth of the community elderly care industry, more talents will be devoted to the industry, and more and more detailed evaluation models can be put forward for community elderly care communications and medical care. In general, the results of this study provide theoretical support for the development of the rehabilitation service model and daily health management of community medical stations for elderly patients and meet the rehabilitation service needs of the majority of elderly groups.

## Figures and Tables

**Figure 1:** The structure of the medical information monitoring system for the elderly in the community. (a) Front-end data collection, (b) wireless data transmission, and (c) background data management.

**Figure 2:** Schematic diagram of photoplethysmography: (A) the light transmission of the human body and (B) the sensor data collection.

**Figure 3:** Working principle of three-axis acceleration sensor: (a) the three-axis detection of the three-axis sensor and (b) the acceleration detection of the three-axis sensor.

**Figure 4:** The first health survey of the elderly population in the community.

**Figure 5:** Results of risk analysis and evaluation of physiological indicators for the elderly.

**Figure 6:** Steps for attribute reduction algorithm. The particle fitness value can be calculated with equation (11).

**Figure 7:** Flowchart for attribute reduction and parameter optimization based on PSO-SVM.

**Figure 8:** Comparison results of fusion algorithms.

**Table 1:** Items for elderly ability assessment.

First-level indicators	Second-level indicators
Behavioral ability	Eating, going to the toilet, walking on level ground, walking on slopes, walking on stairs, picking and placing, moving, hanging and taking, self-care, and exercise
Mental state	Emotional cognition, emotional expression, depressive symptoms, aggression, irritability, and self-awareness
Receive feedback	Listening, speaking, reading, writing, spatial positioning, and level of consciousness
Social participation	Interpersonal communication, activity participation, character identification, and workability

**Table 2:** Risk assessment models for elderly diseases.

Average blood pressure (mmhg)	Risk grade	Pulmonary arterial pressure (mmhg)	Heart rate (time/min)	SpO_2_ (%)	Body temperature (°C)	Breathing rate (time/min)
114	2	26	108	98	36.7	20

**Table 3:** Some elderly physiological indicators in the database.

Average blood pressure (mmhg)	Risk grade	Pulmonary arterial pressure (mmhg)	Heart rate (time/min)	SpO2 (%)	Body temperature (°C)	Breathing rate (time/min)
114	2	26	108	98	36.7	20
112	2	24	102	98	36.8	19
121	2	24	104	99	36.8	18
118	2	27	103	98	36.8	20
116	2	28	105	98	36.7	20
118	2	26	112	98	37.1	22
120	2	29	121	95	37.1	25
102	2	33	132	97	36.9	25

**Table 4:** Characteristic values and contribution rate of sample data.

Eigenvalue	3.6107	1.1032	0.9037	0.2304	0.1425	0.0603

Contribution rate	70.056	16.746	6.8935	3.7425	2.2469	0.8825

## Data Availability

All data included in this study are available upon request by contact with the corresponding author.
